The article "Excision of viral reprogramming cassettes by Cre protein transduction enables rapid, robust and efficient derivation of transgene-free human induced pluripotent stem cells" was published in 2014. Journal: Stem Cell Res Ther.

# Excision of viral reprogramming cassettes by Cre protein transduction enables rapid, robust and efficient derivation of transgene-free human induced pluripotent stem cells

**DOI:** 10.1186/scrt435

**Published:** 2014-04-08

**Authors:** Asifiqbal Kadari, Min Lu, Ming Li, Thileepan Sekaran, Rajkumar P Thummer, Naomi Guyette, Vi Chu, Frank Edenhofer

**Affiliations:** 1 Stem Cell Engineering Group, Institute of Reconstructive Neurobiology, University of Bonn – Life & Brain Center and Hertie Foundation, Sigmund-Freud Straße 25, 53105 Bonn, Germany; 2 EMD-Millipore, Bioscience Division, Stem Cell Group, Temecula, CA 92590, California; 3 Present address: Irvine Pharmaceutical Services, Irvine, CA 92618, USA; 4 Stem Cell and Regenerative Medicine Group, Institute of Anatomy and Cell Biology, Julius-Maximilians-University Würzburg, Koellikerstraße 6, D-97070 Würzburg, Germany

## Abstract

Integrating viruses represent robust tools for cellular reprogramming; however, the presence of viral transgenes in induced pluripotent stem cells (iPSCs) is deleterious because it holds the risk of insertional mutagenesis leading to malignant transformation. Here, we combine the robustness of lentiviral reprogramming with the efficacy of Cre recombinase protein transduction to derive iPSCs devoid of transgenes. By genome-wide analysis and targeted differentiation towards the cardiomyocyte lineage, we show that transgene-free iPSCs are superior to iPSCs before Cre transduction. Our study provides a simple, rapid and robust protocol for the generation of clinical-grade iPSCs suitable for disease modeling, tissue engineering and cell replacement therapies.

## Introduction

Initial reports for generating induced pluripotent stem cells (iPSCs) involved retroviruses as a mode of transgene delivery [1]. Although retroviruses are capable of reprogramming somatic cells to iPSCs, the clinical applicability of such iPSCs is limited due to the integrated transgenes carrying the risk of insertional mutagenesis [2] and tumor formation [3]. Moreover, continuous expression of transgenes in iPSCs negatively affects pluripotency [4] and limits their differentiation potential [5]. These effects have been shown by the inability to yield live chimeric mice and the diminished endodermal differentiation of iPSCs carrying transgenes [5]. Alternative approaches were explored to obtain higher efficiency with minimal genetic modifications of the cells. Various protocols circumventing viral vectors have been published, including the use of transposons [6], episomal plasmids [7], synthetic mRNA [8], microRNAs [9], Sendai virus [10] as well as protein transduction [11-13]. iPSCs generated by these methods contain minimal or no genetic modifications and are generally more suitable for clinical applications than cells derived by virus-based protocols. However, still there is no gold standard for an iPSC reprogramming strategy since these non-integrating approaches exhibit limitations such as low reprogramming efficiencies, slow reprogramming kinetics, a narrow range of cell specificity, and poor reproducibility [14,15]. In terms of robustness and efficacy, therefore, the retroviral and lentiviral system still represents the method of choice for iPSC derivation [16].

Early attempts to improve viral-based iPSC protocols included the use of polycistronic vectors. The core element of those vectors is a cassette, consisting of cDNAs of the four transcription factors, linked together via 2A self-cleaving peptide sequences [17,18]. This strategy allows translation of four separate polypeptides from a single mRNA strand. Thus, instead of four viruses, a single construct is sufficient to induce cellular reprogramming. This approach decreases the risk of insertional mutagenesis. Various biomedical applications of iPSCs will not strictly require cells completely free from genetic modifications. Hence, a Cre-excisable lentiviral system would provide a rapid and easy alternative for the generation of transgene-free iPSC clones. The usage of polycistronic vectors harboring loxP sites allows transgene excision from iPSCs via transient expression of Cre recombinase [19]. However, the reprogramming efficiency using these vectors was reported to be only 0.01% [19]. In 2009 Sommer and colleagues reported an improved lentiviral vector to overcome this limitation by yielding a reprogramming efficiency of 0.1 to 1.5% [20]. Moreover, the vector could also reprogram peripheral blood cells that are usually quite resistant towards reprogramming [21]. However, deletion of the loxP-flanked transgene cassette requires introduction of Cre recombinase activity. This activity has been accomplished by either transfection of iPSCs with a Cre-encoding plasmid [19,22] or using an adenoviral Cre construct [5,23] and subsequent genetic identification of successfully recombined clones. More recently, transgene-free iPSCs were obtained by excising the transgene cassette by delivery of Cre mRNA [24]. However, this protocol involves daily transfection of mRNA for a week to perform excision. This rather inefficient and laborious transfection and selection procedure makes Cre/loxP-based iPSC derivation less appealing for obtaining transgene-free iPSCs. In fact, efficient and reliable induction of Cre recombinase activity in loxP-modified iPSCs and subsequent selection of cleaned clones represents a roadblock for the widespread use of Cre-deletable iPSC systems.

Direct delivery of biologically active Cre protein has been shown to be a highly efficient and robust method for inducing Cre recombinase activity in mammalian cells [25-28]. We reported a cell-permeable recombinant Cre protein that was generated by fusing Cre with the cell-penetrating peptide TAT and a nuclear localization sequence [29]. The TAT peptide confers cell permeability and the nuclear localization sequence targets the fusion protein to the nucleus. TAT-Cre was used for site-specific recombination in human embryonic stem cells (ESCs) with more than 90% recombination efficiency [27]. Here, we show rapid derivation of transgene-free human iPSC clones by combining direct delivery of biologically active TAT-Cre protein with robust reprogramming by a lentiviral polycistronic vector. We demonstrate that transgene deletion renders iPSCs that resemble more human ESCs with respect to gene expression than transgene-harboring cells before deletion. Moreover, we show a strong enhancement of differentiation towards the cardiac lineage in transgene-free iPSCs as compared with loxP-modified iPSCs.

## Materials and methods

### Reprogramming of human fibroblasts and characterization of iPSCs

The human fibroblasts used in this study were obtained from a skin punch biopsy of a 24-year-old male after obtaining informed consent and ethical clearance by the ethics committee of the University of Würzburg, Germany (ethical report number 96/11, dated 10 June 2011). Human fibroblasts were infected with the Human STEMCCA Cre-Excisable constitutive polycistronic (OKSM) lentiviral vector [22] and were seeded on irradiated mouse embryonic fibroblasts in a reprogramming medium consisting of Dulbecco’s modified Eagle’s medium/F12 (Sigma-Aldrich, St. Louis, MO, USA) with 20% KnockOut Serum Replacement (Invitrogen, Carlsbad, CA, USA), 1 mM non-animal l-glutamine (Sigma-Aldrich), 0.1 mM β-mercaptoethanol (Sigma-Aldrich), 1% non-essential amino acids (Invitrogen), and 10 ng/ml basic fibroblast growth factor (Invitrogen). After 3 weeks, iPSC-like colonies were picked, expanded on matrigel-coated dishes and characterized for the pluripotency markers Oct4 (Santacruz Biotechnology, Finnell Street Dallas, Texas 75220 USA) and SSEA-4 (Millipore, Temecula, CA, USA) antibodies.

### TAT-Cre treatment of human iPSCs

Human iPSCs were maintained on matrigel-coated dishes in mTeSR™1 (STEMCELL Technologies, Temecula, CA, USA) or PluriSTEM™ (EMD Millipore, Vancouver, BC, Canada) medium. Human iPSC colonies were treated with alphazyme (1 ml/well in a six-well plate; PAA, Linz, Austria) for 5 to 10 minutes to obtain single cells. Then 100,000 to 200,000 cells were seeded in each well of a six-well plate having mTeSR™1 or PluriSTEM™ medium with 10 μM Rock inhibitor (Y27632; Sigma-Aldrich) to prevent the cell apoptosis. Twenty-four hours later, the medium was changed to mTeSR™1 or PluriSTEM™ containing TAT–Cre (catalogue number SCR508; EMD Millipore) with different concentrations of 0.5 μM, 1 μM and 2 μM. Cells were incubated with TAT-Cre recombinant protein for 5 hours. Cells were grown for 1 week and colonies were expanded either monoclonally or polyclonally, and then polymerase chain reaction (PCR) was performed to assess transgene deletion. Transgene-deleted clones were expanded and characterized further by immunostaining and differentiation.

### Excision of the reprogramming cassette

To confirm the transgene deletion, genomic DNA from TAT-Cre-treated subclones were isolated and PCR was performed with the following conditions: 95°C for 2 minutes; followed by 34 cycles of 94°C for 30 seconds, 60°C for 30 seconds, and 72°C for 45 seconds; followed by a single cycle of 72°C for 5 minutes using the primers WPRE forward, ATCATGCTATTGCTTCCCGTATGGC and WPRE reverse, GGAGATCCGACTCGTCTGAGG, and β-actin forward, GGCTACAGCTTCACCACCAC and β-actin reverse, CCACCTTCCAGCAGATGTGG.

### Immunostaining

For iPSC characterization, immunostaining was performed using Oct4 (1:100; Santacruz Biotechnology) and SSEA-4 (1:200; Millipore) antibodies. Briefly, cells were washed with phosphate-buffered saline (PBS), fixed with 4% paraformaldehyde for 15 minutes and permeabilized in PBS containing 0.1% Triton X-100 and 5% fetal calf serum for 30 minutes. Cells were then incubated overnight with the Oct4 and SSEA-4 antibodies. Next day, secondary antibodies Alexa 488 and Alexa 555 (1:1000; Life Technologies, Carlsbad, CA, USA) were used to detect and visualize the primary antibodies. All antibodies were diluted in blocking solution. Micrographs were taken with an Axiovert 200 M microscope (Carl Zeiss, Oberkochen, Badenwürttemberg, Germany). The above immunostaining protocol was also performed to characterize cardiomyocytes using cardiac Troponin T (cTNT, 1:100; Abcam, Cambridge, England) and α-actinin (1:200; Sigma-Aldrich) as a primary antibody and Alexa 488 as a secondary antibody.

### Teratoma formation and karyotype analysis

Pluripotency was tested by injection of the test cell population into the testes of immune-deficient NOD/SCID mice. Then 0.5 × 10^6^ to 5 × 10^6^ cells were injected using a pulled glass capillary pipette that was advanced via the efferent ducts through the rete testis into the interstitial space of the testis. Animals were euthanized when palpable tumors were present or at 4 months after injection, whichever came first. The teratomas were fixed in 10% neutral buffered formalin, dehydrated (graded alcohols), cleared (xylene) and embedded with paraffin wax (formalin fixed paraffin embedded). Then 5 μm sections were cut, floated on a water bath and picked up on positively charged slides (Probe On Plus). Sections were then deparaffinized in three changes of xylene, rehydrated in a series of graded alcohols (100% × 2, 70% × 2, 30% × 2, distilled H_2_O × 2) and hematoxylin and eosin staining was performed. Karyotype analysis was performed on 20 G-banded metaphase cells for TAT-Cre excised human iPSC clone at p13 by Cell Line Genetics (Madiso, WI, USA).

### Gene expression analysis

RNA was isolated using the RNeasy-Kit (Qiagen, Hilden, Germany). mRNA transcription levels were evaluated using the Human HT-12 array (version 4, revision 2; Qiagen, Hilden, Germany), which consists of 47,323 probes and described mRNA features. All samples were processed at least in duplicate to reduce signals arising from processing artifacts. Data processing was performed using the GenomeStudio suite version 2011.1 and the Gene expression module version 1.9.4 (both Illumina Inc., San Diego, CA, USA). Gene expression data analysis was carried out with the R and Bioconductor packages, and their intensities were quantile normalized. The differentially expressed genes were determined by applying the empirical Bayes test statistics, and the Benjamini–Hochberg false discovery method was used for multiple testing correction. Genes with fold-change >2 and *P* ≤ 0.5 were considered differentially expressed and were used for subsequent analysis. The data discussed in this publication have been deposited in the National Center for Biotechnology Information Gene Expression Omnibus [GEO:GSE55725].

### Generation of the Cre reporter human iPSC line

Human iPSC line del-AR1034ZIMA (del-ARiPS) clone 1.4 was treated with alfazyme to obtain a single-cell suspension. Then 200,000 cells were seeded in one well of a six-well plate in mTeSR™1 medium with 10 μM Rock inhibitor. On the next day, cells were infected with lentivirus containing EF1α-Cre reporter–puromycin construct (modified from original construct [30] by replacing CMV promoter by EF1α promoter). Forty-eight hours later, the medium was changed to mTeSR™1 with puromycin (1 μg/ml) for 5 days to obtain colonies with stably integrated Cre reporter construct.

### Cardiomyocyte differentiation of human iPSCs

Human iPSCs were maintained on matrigel-coated plates in mTeSR™1 medium until they reached 80% confluency. Cardiac differentiation was induced by Activin A (5 ng/ml), BMP4 (25 ng/ml) and Chir99021 (5 μM) in RPMI 1640 medium containing B27 and 2 mM glutamine as a basal medium for 3 days. From day 4, cells were kept in basal medium containing Wnt inhibitor XAV939 for 5 days followed by further culture in basal medium.

### Flow cytometry

Cells (1 × 10^6^) were trypsinized and fixed with 4% paraformaldehyde for 10 minutes. Cells were then washed with PBS, permeabilized in PBS containing 0.1% Triton X-100 and 5% fetal calf serum for 30 minutes and incubated for 2 hours with cTNT antibody (1:100; Abcam). No antibody was taken as a negative control. Cells were then washed once with PBS containing 0.1% Tween-20 and resuspended in PBS containing 0.1% Triton-X 100 and 5% fetal calf serum and secondary antibody Alexa 488 anti-mouse IgG (1:1,000; Life Technologies) for 1 hour in the dark. Finally, cells were washed again with PBS containing 0.1% Tween-20 and measured for FACS analysis. Analysis was performed by the Flow Jo program.

## Results

### Overview of generation of transgene-free human iPSCs with TAT-Cre application

Previous studies have shown successful derivation of transgene-free iPSCs by excising a loxP-flanked transgene cassette with Cre plasmid [19], Adeno-Cre [5,23] or Cre mRNA [24]. We aimed at improving this approach by employing Cre protein transduction to enhance the efficiency as well as to accelerate the process of obtaining transgene-free iPSCs. Our protocol does not require repeated transfections or viral preparations (see schematic overview in Figure 1). To generate human iPSCs we utilized the lentiviral vector STEMCCA, which was shown to be more efficient [20] than earlier Cre-excisable lentiviral vectors [19]. We infected human dermal fibroblasts and obtained the AR1034ZIMA loxP-modified iPSC line (fl-ARiPS). As described in the scheme, we treated a single cell suspension of fl-ARiPS cells with a single application of TAT-Cre recombinant protein. TAT-Cre-treated cells were expanded either monoclonally or polyclonally to yield transgene-excised iPSCs ready for further analyses (Figure 1B). For the confirmation of transgene excision, PCR against the viral WPRE element was used (Figure 1C).

**Figure 1:** **Scheme of induced pluripotent stem cell generation and subsequent Cre protein transduction to obtain transgene-free induced pluripotent stem cells. (A)** Reprogramming of human fibroblasts to induced pluripotent stem cells (iPSCs) via lentiviral vector STEMCCA. **(B)** Schematic representation of TAT-Cre treatment to obtain transgene-free iPSCs. **(C)** Schematic representation of the genomic locus before (top) and after (bottom) Cre-mediated recombination. LTR, long terminal repeat; PCR, polymerase chain reaction.

### Assessment of TAT-Cre-mediated transgene deletion efficiency

First, we used Cre protein transduction conditions that we elaborated for Cre-mediated excision in human ESCs cultivated on mouse feeder cells [27]. Moreover, to make it practically more feasible we adopted our iPSC lines to feeder-free conditions, which we assumed to result in higher transgene deletion efficiency with a lower concentration of TAT-Cre. In particular, we prepared a single cell suspension of fl-ARiPSCs by treating them with alfazyme and seeded them on matrigel-coated plates. Twenty-four hours later, cells were treated with different concentrations of TAT-Cre for 1 to 5 hours. TAT-Cre-treated fl-ARiPS monoclones were expanded and analyzed for transgene deletion. All three monoclones analyzed that were treated with 2 μM TAT-Cre showed excision of the transgene, while in the case of 0.5 and 1 μM TAT-Cre treatment we observed one and two deleted clones, respectively (Figure 2A). To explore the possibility of deletion and subsequent polyclonal cell expansion, we treated the loxP-modified iPSCs with 0.5, 1 and 2 μM TAT-Cre for 5 hours and expanded them polyclonally. Genomic PCR analysis revealed a faint band in the cases of 0.5 and 1 μM, and no band was observed after treatment with 2 μM TAT-Cre, indicating a high excision efficiency that was consistent with the monoclonal analysis (Figure 2B) and previously reported results employing human ESCs [27]. In order to validate the PCR results we mixed genomic DNA from loxP-modified and transgene-deleted iPSC clones in a standardized manner representing corresponding deletion efficiencies. PCR analysis of this dilution series yielded a faint band even in the case of a 99% mixture, while no band was observed with 100% deleted DNA (Figure 2C). Protein transduction was repeated with seven monoclones treated with 1.5, 3 and 6 μM TAT-Cre in each case. As listed in Figure 2D, all clones analyzed showed the deletion of transgenes. Increasing concentrations of TAT-Cre beyond 3 μM resulted in significant cell death and affected the recovery of iPSC colonies after the treatment (data not shown). Upon using higher concentrations of TAT-Cre, excessive cell death was prevented by shortening the time duration of TAT-Cre treatment (5 μM TAT-Cre for 1 hour) without compromising the recombination efficiency. We obtained seven transgene-free clones out of 12 clones tested (Figure 2D). To further confirm the efficiency of TAT-Cre, we monitored the recombination event by integrating a double fluorescence Cre reporter cassette through lentiviral transduction of fl-ARiPSC. We observed more than 95% of cells showing GFP expression with 2 μM TAT-Cre for 5 hours (Figure 2E), confirming the high recombination efficiency determined by PCR analyses.

**Figure 2:** **Assessment of TAT-Cre-mediated transgene deletion efficiency. (A)** Genomic polymerase chain reaction (PCR) for the confirmation of transgene deletion. Three individual clones were treated with 0.5, 1 or 2 μM TAT-Cre for 5 hours and PCR was performed using primers against WPRE and β-actin. F, AR1034ZIMA loxP-modified iPSC line clone 1 (fl-ARiPSC); NC, negative (water) control; WPRE, viral element; BA, β-actin. **(B)** Genomic PCR for the confirmation of transgene deletion in a polyclonal population. fl-ARiPSCs were treated with 0.5, 1 or 2 μM TAT-Cre for 5 hours. Cells were expanded polyclonally and PCR was performed using primers against WPRE and β-actin. **(C)** Validation of genomic PCR analysis. Genomic DNA from loxP-modified and transgene deleted cells were mixed to create defined dilutions as given. **(D)** Quantification of transgene-deleted clones using different concentrations and time duration of TAT-Cre. **(E)** ARiPS-Cre reporter cell line was treated with 2 μM Cre protein to validate recombination efficiency. Cre-mediated recombination induced the expression of green fluorescence protein (EGFP), by deleting the loxP-flanking RFP gene. Scale bar: 120 μm.

### Characterization of transgene-free iPSCs

To assess the pluripotency status of excised del-ARiPS clones, cells were expanded until passage 15 and stained with pluripotency-associated markers Oct4 and SSEA-4. Cells stained positive for both nuclear Oct4 and cell surface marker SSEA-4 (Figure 3A). Furthermore, we performed genome-wide gene expression profiling on del-ARiPS cells and fl-ARiPS cells by microarray analysis. The gene expression datasets were subjected to the recently published bioinformatics assay PluriTest [31] to assess the pluripotency status of reprogrammed cells. According to this analysis, both fl-ARiPS cells and del-ARiPS cells cluster with human ESC line HES I3 in the red-colored background, indicating pluripotency, while fibroblasts are located in the blue region, confirming their nonpluripotent nature (Figure 3B). Notably, del-ARiPS cells appear slightly more shifted to the HES I3 cells as compared with fl-ARiPS cells. Expression profiling of pluripotency-associated genes Oct4, Sox2 and Rex1 as well as fibroblast genes Thy1 and Col5a2 showed similar expression pattern across the iPSCs and human ESCs. Again del-ARiPS cells appear more similar to HES I3 than fl-ARiPS cells (Figure 3C). In fact, there are 63 differentially expressed genes between HES I3 and del-ARiPS cells as compared with more than 130 genes in the case of the parental fl-ARiPS clone (Figure 3D). Furthermore, excised clone could give rise to teratoma consisting of all three germ layers, confirming its *in vivo* differentiation potential (Figure 3E), and showed no chromosomal aberrations as judged by karyotype analysis (Figure 3F).

**Figure 3:** **Characterization of transgene-free induced pluripotent stem cells. (A)** Pluripotency analysis of transgene-excised clones. del-ARiPSCs stain positive for pluripotency-associated markers Oct4 and SSEA-4. Scale bar: 40 μm. **(B)** PluriTest analysis of HES I3, fl-ARiPSC, del-ARiPSC cells and parental fibroblasts to assess pluripotency induction. Cells are distributed based on pluripotency and novelty scores, as indicated by color density background. Red, pluripotency; blue, nonpluripotency. **(C)** Heat-map representation of pluripotency and fibroblast-specific markers. Expression of pluripotency-associated markers Oct4, Sox2 and Rex1 and fibroblast specific markers Thy1 and Col5a2 in induced pluripotent stem cells (iPSCs) and human embryonic stem cells (ESCs) used for this study. **(D)** Venn diagram showing differentially expressed genes. Comparison of differentially expressed genes amongst HES I3, fl-ARiPSC and del-ARiPSC cells. **(E)** Histological analysis of teratoma analysis of excised clone. Teratoma analysis after injection of the excised clone into SCID mice showed formation of all three germ layers: ectoderm (primitive neuroepithelium), mesoderm (cartilage, muscle) and endoderm (glands). **(F)** Karyotype analysis of transgene-excised clone. Cytogenetic analysis on G-banded metaphase cells from excised clone (p13) and all 20 cells demonstrated a normal male karyotype. HES I3, human ESC I3 line; fl-ARiPS, fl-ARiPS iPSC clone 1; del-ARiPS, transgene-free daughter clones of ARIPS iPSC clone 1.

### Improved cardiac differentiation potential of transgene-free iPSCs

To explore whether the deletion of transgenes not only results in genome-wide transcriptional differences but also has functional consequences, we analyzed the differentiation potential by differentiation into the cardiac lineage. To achieve cardiac differentiation, we modified the protocol described by Carpenter and colleagues [32] with the inclusion of modulation of the Wnt signaling pathway using Chir99021 to enhance cardiac differentiation. We employed this protocol for the cardiac differentiation of fl-ARiPS cells and a polyclonal TAT-Cre-treated daughter cell population (2 μM TAT-Cre for 5 hours) (Figure 4A,B). We decided to perform polyclonal expansion in order to reduce the time duration of the entire procedure and to check whether it is possible to see the overall enhancement in differentiation capacity of a polyclonal TAT-Cre-treated population. Indeed, flow cytometry analysis using cTNT as a cardiomyocyte-specific marker indicates a strongly increased differentiation capability of del-ARiPS cells. More than 55% of differentiated del-ARiPS cells are cTNT-positive, whereas only 37% of the parental fl-ARiPSC cells stained positive for cTNT (Figure 4C).

**Figure 4:** **Improved cardiac differentiation potential of transgene-free induced pluripotent stem cells. (A)** Genomic polymerase chain reaction (PCR) for the confirmation of transgene deletion. fl-ARiPS clone 1 was treated with 2 μM TAT-Cre for 5 hours and PCR was performed using primers against WPRE and β-actin (BA). **(B)** Cardiomyocyte differentiation of iPSCs. fl-ARiPS clone 1 and its TAT-Cre-treated polyclonal cell progeny were differentiated towards cardiomyocyte lineage using cardio-inductive medium. Cells were stained with α-actinin antibody at day 15. Scale bar: 40 μm. **(C)** Flow cytometry analysis of cardiac-specific troponin T (cTNT) staining at day 15 of cardiac differentiation. Cardiac differentiation showed an increase from 37 to 56% cTNT-positive cardiomyocytes in the case of TAT-Cre-treated cell populations. The experiment was repeated twice with similar results.

## Discussion

In this study we demonstrate an efficient way of obtaining iPSCs with minimal genetic modifications by combining the widely applied and robust lentiviral reprogramming approach with the highly efficient and less invasive TAT-Cre-mediated transgene deletion. Earlier studies have reported the deletion of transgenes by delivering Cre as a plasmid, as Adeno-Cre, or by mRNA transfection [5,19,22-24]. The protocol elaborated by Soldner and colleagues yielded only 16 transgene-deleted clones out of 180 analyzed after transfecting iPSCs with a Cre-encoding plasmid and subsequent selection either with green fluorescent protein fluorescence or puromycin [19]. The relatively low efficiency might be due to the transient transfection of Cre, which is limiting intracellular DNA recombinase activity. Sommer and colleagues and Somers and colleagues used Adeno-Cre and Cre-IRES-Puro constructs respectively to achieve higher excision efficiencies [5,22]. A more recent study by Awe and colleagues demonstrate transgene excision in iPSC clones with putative clinical grade status using Adeno-Cre-mediated transgene deletion. During their transgene excision analysis the authors obtained only one transgene-excised subclone out of six Adeno-Cre-treated clones [23]. Furthermore, deletion approaches using Cre plasmids or Adeno-Cre constructs require transfection and subsequent selection of cells with Cre recombinase activity either by flow cytometry sorting or by antibiotic selection. Such relatively complicated steps are undesirable because they might be stressful to the cells [33]. Moreover, there is the possibility that Cre-encoding plasmids or viral constructs integrate into the genome [34]. More recently, the group of George Daley has reported transgene excision by transfecting loxP-modified iPSC with Cre-encoding mRNA. Notably, this procedure involves daily transfections of Cre mRNA for 4 hours up to 7 days, which again represents a complicated and stressful procedure for the cells. The protocol developed in our study, in contrast, requires just a single application of TAT-Cre recombinant protein for 5 hours due to its high recombination efficiency. By this, the use of TAT-Cre accelerates the process of obtaining transgene-free iPSCs with minimal technical complexity. During our analysis, transgene-free iPSCs remain pluripotent. Moreover, microarray analysis indicates enhancement in the quality of iPSCs, as transgene-excised iPSCs are more similar to human ESCs with respect to gene expression profiling, confirming previous studies [19]. In fact, transgene-free iPSCs exhibit an improved differentiation potential [5]. In our study, we show enhanced cardiac differentiation of TAT-Cre-treated polyclonal iPSCs. By this we show an improvement in differentiation capacity of a polyclonal cell population after the removal of transgenes with Cre-mediated recombination. This makes TAT-Cre protein an attractive tool to obtain transgene-free iPSCs even in a polyclonal manner as recently suggested [35], circumventing the laborious selection procedure of transgene-excised clones. In conclusion, our study provides a simple, rapid and robust protocol for the generation of superior transgene-free iPSCs suitable for disease modeling, drug and toxicity screening, as well as cell replacement therapies.

## Conclusions

In summary, our study outlines efficient derivation of factor-free human iPSC lines by combinatorial use of the robust lentivirus human STEMCCA vector and highly efficient TAT-Cre protein transduction. We have shown enhanced quality of transgene-free iPSCs using microarray analysis and cardiac differentiation. Moreover, we show polyclonal expansion of transgene-deleted clones that circumvents laborious selection procedures and time-consuming analysis of subclones.

## Abbreviations

cTNT: cardiac Troponin T; del-ARiPS: AR1034ZIMA transgene-free daughter clones of ARIPS iPSC clone 1; fl-ARiPS: AR1034ZIMA loxP-flanked transgene ARiPS iPSC clone 1; HES I3: human ESC I3 line; ESC: embryonic stem cell; iPSC: induced pluripotent stem cell; PBS: phosphate-buffered saline; PCR: polymerase chain reaction.

## Competing interests

MLu, MLi, NG and VC are salaried employees at EMD Millipore. The remaining authors declare that they have no competing interests.

## Authors’ contributions

AK was responsible for the conception, design, collection and/or assembly of data, data analysis, interpretation, manuscript writing, and final approval of the manuscript. MLu, MLi, NG, VC and TS collected and/or assembled data. RPT performed data analysis and manuscript writing. FE was responsible for conception and design, financial support, collection and/or assembly of data, data analysis and interpretation, manuscript writing, and final approval of manuscript. All authors contributed to the final draft of the manuscript.

## References

[B1] TakahashiKYamanakaSInduction of pluripotent stem cells from mouse embryonic and adult fibroblast cultures by defined factorsCell200612666367610.1016/j.cell.2006.07.02416904174

[B2] MikkersHBernsARetroviral insertional mutagenesis: tagging cancer pathwaysAdv Cancer Res20038853991266505310.1016/s0065-230x(03)88304-5

[B3] OkitaKIchisakaTYamanakaSGeneration of germline-competent induced pluripotent stem cellsNature200744831331710.1038/nature0593417554338

[B4] KoppJLOrmsbeeBDDeslerMRizzinoASmall increases in the level of Sox2 trigger the differentiation of mouse embryonic stem cellsStem Cells20082690391110.1634/stemcells.2007-095118238855

[B5] SommerCASommerAGLongmireTAChristodoulouCThomasDDGostissaMAltFWMurphyGJKottonDNMostoslavskyGExcision of reprogramming transgenes improves the differentiation potential of iPS cells generated with a single excisable vectorStem Cells20102864741990483010.1002/stem.255PMC4848036

[B6] KajiKNorrbyKPacaAMileikovskyMMohseniPWoltjenKVirus-free induction of pluripotency and subsequent excision of reprogramming factorsNature200945877177510.1038/nature0786419252477PMC2667910

[B7] ChouBKMaliPHuangXYeZDoweySNResarLMZouCZhangYATongJChengLEfficient human iPS cell derivation by a non-integrating plasmid from blood cells with unique epigenetic and gene expression signaturesCell Res20112151852910.1038/cr.2011.1221243013PMC3193421

[B8] WarrenLManosPDAhfeldtTLohYHLiHLauFEbinaWMandalPKSmithZDMeissnerADaleyGQBrackASCollinsJJCowanCSchlaegerTMRossiDJHighly efficient reprogramming to pluripotency and directed differentiation of human cells with synthetic modified mRNACell Stem Cell2010761863010.1016/j.stem.2010.08.01220888316PMC3656821

[B9] Anokye-DansoFTrivediCMJuhrDGuptaMCuiZTianYZhangYYangWGruberPJEpsteinJAMorriseyEEHighly efficient miRNA-mediated reprogramming of mouse and human somatic cells to pluripotencyCell Stem Cell2011837638810.1016/j.stem.2011.03.00121474102PMC3090650

[B10] FusakiNBanHNishiyamaASaekiKHasegawaMEfficient induction of transgene-free human pluripotent stem cells using a vector based on Sendai virus, an RNA virus that does not integrate into the host genomeProc Jpn Acad Ser B Phys Biol Sci20098534836210.2183/pjab.85.34819838014PMC3621571

[B11] BosnaliMEdenhoferFGeneration of transducible versions of transcription factors Oct4 and Sox2Biol Chem20083898518611868182610.1515/BC.2008.106

[B12] KimDKimCHMoonJIChungYGChangMYHanBSKoSYangEChaKYLanzaRKimKSGeneration of human induced pluripotent stem cells by direct delivery of reprogramming proteinsCell Stem Cell2009447247610.1016/j.stem.2009.05.00519481515PMC2705327

[B13] ZhouHWuSJooJYZhuSHanDWLinTTraugerSBienGYaoSZhuYSiuzdakGSchölerHRDuanLDingSGeneration of induced pluripotent stem cells using recombinant proteinsCell Stem Cell2009438138410.1016/j.stem.2009.04.00519398399PMC10182564

[B14] GonzalezFBoueSIzpisua BelmonteJCMethods for making induced pluripotent stem cells: reprogramming a la carteNat Rev Genet2011122312422133976510.1038/nrg2937

[B15] WorsdorferPThierMKadariAEdenhoferFRoadmap to cellular reprogramming – manipulating transcriptional networks with DNA, RNA, proteins and small moleculesCurr Mol Med2011138688782364206710.2174/1566524011313050017

[B16] SommerCAMostoslavskyGExperimental approaches for the generation of induced pluripotent stem cellsStem Cell Res Ther201012610.1186/scrt2620699015PMC2941118

[B17] CareyBWMarkoulakiSHannaJSahaKGaoQMitalipovaMJaenischRReprogramming of murine and human somatic cells using a single polycistronic vectorProc Natl Acad Sci U S A200910615716210.1073/pnas.081142610619109433PMC2629226

[B18] SzymczakALWorkmanCJWangYVignaliKMDilioglouSVaninEFVignaliDACorrection of multi-gene deficiency in vivo using a single ‘self-cleaving’ 2A peptide-based retroviral vectorNat Biotechnol20042258959410.1038/nbt95715064769

[B19] SoldnerFHockemeyerDBeardCGaoQBellGWCookEGHargusGBlakACooperOMitalipovaMIsacsonOJaenischRParkinson’s disease patient-derived induced pluripotent stem cells free of viral reprogramming factorsCell200913696497710.1016/j.cell.2009.02.01319269371PMC2787236

[B20] SommerCAStadtfeldMMurphyGJHochedlingerKKottonDNMostoslavskyGInduced pluripotent stem cell generation using a single lentiviral stem cell cassetteStem Cells20092754354910.1634/stemcells.2008-107519096035PMC4848035

[B21] StaerkJDawlatyMMGaoQMaetzelDHannaJSommerCAMostoslavskyGJaenischRReprogramming of human peripheral blood cells to induced pluripotent stem cellsCell Stem Cell20107202410.1016/j.stem.2010.06.00220621045PMC2917234

[B22] SomersAJeanJCSommerCAOmariAFordCCMillsJAYingLSommerAGJeanJMSmithBWLafyatisRDemierreMFWeissDJFrenchDLGaduePMurphyGJMostoslavskyGKottonDNGeneration of transgene-free lung disease-specific human induced pluripotent stem cells using a single excisable lentiviral stem cell cassetteStem Cells2010281728174010.1002/stem.49520715179PMC3422663

[B23] AweJPLeePCRamathalCVega-CrespoADurruthy-DurruthyJCooperAKarumbayaramSLowryWEClarkATZackJASebastianoVKohnDBPyleADMartinMGLipshutzGSPhelpsPEPeraRAByrnJAGeneration and characterization of transgene-free human induced pluripotent stem cells and conversion to putative clinical-grade statusStem Cell Res Ther201348710.1186/scrt24623890092PMC3854769

[B24] LohYHYangJCDe Los AngelesAGuoCCherryARossiDJParkIHDaleyGQExcision of a viral reprogramming cassette by delivery of synthetic Cre mRNACurr Protoc Stem Cell Biol2012Chapter 4Unit4A 52260564810.1002/9780470151808.sc04a05s21PMC3397830

[B25] PatschCEdenhoferFConditional mutagenesis by cell-permeable proteins: potential, limitations and prospectsHandb Exp Pharmacol200717820323210.1007/978-3-540-35109-2_917203657

[B26] HauptSEdenhoferFPeitzMLeinhaasABrustleOStage-specific conditional mutagenesis in mouse embryonic stem cell-derived neural cells and postmitotic neurons by direct delivery of biologically active Cre recombinaseStem Cells20072518118810.1634/stemcells.2006-037116960133

[B27] NoldenLEdenhoferFHauptSKochPWunderlichFTSiemenHBrustleOSite-specific recombination in human embryonic stem cells induced by cell-permeant Cre recombinaseNat Methods2006346146710.1038/nmeth88416721380

[B28] PeitzMJagerRPatschCJagerAEgertASchorleHEdenhoferFEnhanced purification of cell-permeant Cre and germline transmission after transduction into mouse embryonic stem cellsGenesis20074550851710.1002/dvg.2032117661398

[B29] PeitzMPfannkucheKRajewskyKEdenhoferFAbility of the hydrophobic FGF and basic TAT peptides to promote cellular uptake of recombinant Cre recombinase: a tool for efficient genetic engineering of mammalian genomesProc Natl Acad Sci U S A2002994489449410.1073/pnas.03206869911904364PMC123675

[B30] RussHABarYRavassardPEfratSIn vitro proliferation of cells derived from adult human beta cells revealel by cell lineage tracingDiabetes2008571575158310.2337/db07-128318316362

[B31] MullerFJSchuldtBMWilliamsRMasonDAltunGPapapetrouEPDannerSGoldmannJEHerbstASchmidtNOAldenhoffJBLaurentLCLoringJFA bioinformatic assay for pluripotency in human cellsNat Methods2011831531710.1038/nmeth.158021378979PMC3265323

[B32] CarpenterLCarrCYangCTStuckeyDJClarkeKWattSMEfficient differentiation of human induced pluripotent stem cells generates cardiac cells that provide protection following myocardial infarction in the ratStem Cells Dev20122197798610.1089/scd.2011.007522182484PMC3315757

[B33] MoranDMShenHMakiCGPuromycin-based vectors promote a ROS-dependent recruitment of PML to nuclear inclusions enriched with HSP70 and ProteasomesBMC Cell Biol2009103210.1186/1471-2121-10-3219409099PMC2685373

[B34] GloverDJLippsHJJansDATowards safe, non-viral therapeutic gene expression in humansNat Rev Genet2005629931010.1038/nrg157715761468

[B35] WillmannCAHemedaHPieperLALenzMQinJJoussenSSontagSWanekPDeneckeBSchulerHMZenkeMWagnerWTo clone or not to clone? Induced pluripotent stem cells can be generated in bulk culturePLoS One20138e6532410.1371/journal.pone.006532423734247PMC3667031

